# Clinical Analysis of Video-Assisted Thoracoscopic Surgery for Resection of Solitary Pulmonary Nodules and Influencing Factors in the Diagnosis of Benign and Malignant Nodules

This article has been retracted.

**DOI:** 10.1155/2021/1490709

**Published:** 2021-08-30

**Authors:** Hongxu Yue, Kaijie Fan, Zhimin Zhang, Yang Liu

**Affiliations:** ^1^Postgraduate School, Medical School of Chinese PLA, Beijing 100853, China; ^2^Department of Thoracic Surgery, The First Medical Center of Chinese PLA General Hospital, Beijing 100853, China; ^3^Department of Thoracic Surgery, The Third Medical Center of Chinese PLA General Hospital, Beijing 100089, China

## Abstract

**Purpose:**

This is a retrospective research comparing the clinical outcomes of single-hole versus multi-hole video-assisted thoracoscopic surgical (VATS) resection for solitary pulmonary nodules (SPN) and examining the factors influencing the diagnosis of benign and malignant pulmonary nodules.

**Method:**

We collected the clinical data, surgical status, outcomes, and corresponding imaging features of 317 patients with SPN who were surgically resected by VATS and diagnosed as benign or malignant by pathology in our hospital from January 2019 to December 2021.

**Result:**

Among the 317 patients, 124 (39.12%) underwent single-port VATS and 193 (60.88%) underwent multiple-hole VATS. All patients were grouped according to the different surgical methods, and their postoperative indicators were statistically analyzed. The results showed that neither the single-port VATS group nor the multi-port VATS group had any serious adverse events such as death during the perioperative period. The average operation time, intraoperative blood loss, drainage tube indwelling time, and postoperative hospital stay were significantly lower in the two groups. Statistics of postoperative pathological diagnosis showed that 98 cases (30.91%) of all nodules were benign nodules and 219 cases (69.09%) were malignant nodules, and a further single-multivariate analysis showed that age, nodule maximum diameter, lobular sign, burr sign, vascular cluster sign, and pleural depression sign were independent relevant factors for the diagnosis of benign and malignant nodules.

**Conclusion:**

VATS is less invasive and has fewer complications and is of great clinical value for both diagnosis and treatment of benign and malignant SPN. Age, maximum nodal diameter, lobar sign, burr sign, vascular set sign, and pleural depression sign were independent correlates affecting the diagnosis of benign and malignant SPN, which reminds that great attention should be paid to patients who are older and have risk factors on imaging, and early and timely active treatment or close follow-up should be carried out.

## 1. Introduction

Solitary pulmonary nodules (SPNs) are round or round-like lesions ≤30 mm in diameter within the lung parenchyma and are not associated with significant pulmonary atelectasis, satellite lesions, pleural effusion, or lymph node enlargement [1]. The detection rate of SPN is showing an increasing trend with the improvement of people's awareness of physical examination and the development of imaging technology. The emergence of SPN is often a sign of lung metastasis of early lung cancer or other malignant tumors and needs to be removed in time to avoid delaying the disease. However, early diagnosis can avoid unnecessary surgery for benign SNP [2]. It can be seen that early diagnosis of SPN and selection of the best treatment plan in the process of clinical practice are important ways to treat patients with lung tumors and reduce their mortality.

The diagnosis and differentiation of isolated pulmonary nodules is difficult, and the combination of imaging and pathology, such as magnetic resonance imaging (MRI), computer tomography (CT), and X-ray, is often used in clinical practice to implement the diagnosis and management, but there is not a high positive detection rate [3]. The open-chest surgical exploration operation is a common and practical intraoperative diagnostic method, but this procedure can cause greater trauma to the patient's body and is prone to various postoperative complications such as lung infection. In addition, open-heart surgery usually takes a long time, which increases the risk of surgery and requires a long postoperative period of intrathoracic drainage, which has a serious impact on the patient's quality of life and is not conducive to early recovery [4, 5]. Video-assisted thoracoscopic surgery (VATS) surgical approach is less traumatic, with fewer postoperative complications, avoiding additional nerve and tissue damage to the patient, and better postoperative rehabilitation, and diagnosis and treatment can be performed at the same time. The patient does not need to undergo a second operation, which reduces the burden on the patient to a greater extent and avoids repeated inspections and delays in treatment [6, 7]. In this study, we retrospectively analyzed 317 cases of SPN patients undergoing VATS surgical resection and pathological diagnosis of benign and malignant SPN in our hospital and explored the efficacy of VATS and related factors affecting the diagnosis of benign and malignant SPN.

## 2. Materials and Methods

### 2.1. General Information

The clinical data of 317 patients with SPN who were surgically resected by VATS and confirmed benign and malignant by pathology at our hospital from January 2017 to December 2019 were retrospectively analyzed. Among them, 176 males and 141 females were aged from 38 to 70 years, and the average age was (54.83 ± 10.29) years. There were 68 patients who had symptoms of cough and sputum; 89 patients had symptoms such as chest tightness, chest pain, and low-grade fever; and 164 patients had no abnormal symptoms and SPN were found through health examination. There were 127 cases with a history of smoking and 26 cases with a history of previous tumors, and the maximum diameter of the nodule was (22.81 ± 5.34) mm. There were 96 cases in the right upper lobe, 31 cases in the right middle lobe, 58 cases in the right lower lobe, 79 cases in the left upper lobe, and 53 cases in the left lower lobe according to the classification of the lesion.

### 2.2. Inclusion Criteria

(i) The maximum diameter of SPN is ≤30 mm. (ii) The patient's clinical surgery, pathological data or imaging follow-up data are complete. (iii) The patient has no symptoms such as pleural effusion, obstructive pneumonia, satellite lesions, or hilar mediastinal lymphadenopathy.

### 2.3. Surgical Methods

The patient's routine clinical examination data and chest CT enhanced examination data were sorted out before surgery. The patients were placed in a 90° lying position on the contralateral side when performing VATS. Double-lumen endotracheal intubation was performed, and the contralateral side was used for single-lung ventilation. The surgical method of single-port VATS was as follows: A small 3 cm incision was taken at the mid-axillary line of the fifth intercostal space, and the operations such as insertion of a thoracoscope and all surgical instruments were passed through this hole. In the porous VATS, a 1.2 cm incision was taken from the mid-axillary line of the seventh intercostal space as the observation hole, and a thoracoscope was inserted. A 3-4 cm incision was made between the anterior axillary line and the mid-axillary line of the fourth intercostal space on the surgical side as the operating hole, and surgical instruments were inserted. For patients who have had a pathological diagnosis of malignant tumors before surgery, segmentectomy, lobectomy, or wedge resection was performed according to their lung function, and the corresponding regional lymph nodes were cleared. Lung wedge resection should be performed first, and a quick frozen pathological examination should be done for patients who have no pathological diagnosis before surgery. Then, choose whether to perform lobectomy and lymph node dissection according to the benign and malignant results of the lesion after the frozen pathological report during the operation.

### 2.4. Observation Index

The surgical resection of all patients and the differences in postoperative conditions such as operative time, intraoperative blood loss, chest drain retention time, postoperative hospital stay, and complication rate between patients undergoing single-port VATS and multi-port VATS were observed and recorded. Logistic regression models were used to analyze the factors associated with the diagnosis of benign and malignant SPN.

### 2.5. Statistical Methods

All data were processed with SPSS 22.0 statistical software, and GraphPad Prism 8 was used to make statistical graphs. Measurement data were expressed as mean ± standard deviation ($\bar{x}$ ± *s*), the independent sample t-test was used for comparison between groups, count data were expressed as [*n* (%)], and the chi-square (*χ*^2^) test was performed. A multivariate logistic regression model was used to analyze the related factors affecting the diagnosis of benign and malignant SPN. The difference was statistically significant when *P* < 0.05.

## 3. Results

### 3.1. Surgical Status of Patients

Among the 317 patients, 195 cases (61.51%) underwent lobectomy, 16 cases (5.05%) underwent anatomical segment resection, and 106 cases (33.44%) underwent pulmonary wedge resection. 124 cases (39.12%) underwent single-port VATS, and 193 cases (60.88%) underwent multi-port VATS. During the operation, 3 cases were converted to thoracotomy due to pleural atresia (Figures 1(a) and 1(b)).

### 3.2. Comparison of the Postoperative Situation of Patients Undergoing Single-Port VATS Operation and Multi-Port VATS Operation

All patients were divided into two groups according to the different surgical methods: single-port VATS group and multi-port VATS group. The results showed that there was no significant difference between the two groups in operation time, intraoperative blood loss, thoracic drainage tube indwelling time, postoperative hospital stay, and complication rate (*P* > 0.05, Figures 2(a)–2(e)).

### 3.3. Postoperative Pathological Diagnosis Results of Patients

Among 317 patients, there were 98 benign nodules (30.91%) and 219 malignant nodules (69.09%). The 98 cases of benign nodules included 12 cases of hamartoma, 37 cases of inflammatory pseudotumor, 32 cases of tuberculoma, 2 cases of bronchogenic cyst, 9 cases of sclerosing hemangioma, and 6 cases of solitary fibroma. The 219 cases of malignant nodules included 107 cases of squamous cell carcinoma, 98 cases of adenocarcinoma, 1 case of carcinoid, 2 cases of small cell carcinoma, 8 cases of large cell carcinoma, 2 cases of adenosquamous carcinoma, and 1 case of sarcomatoid carcinoma. The results of TNM staging of malignant nodules were 61 cases in stage IA, 72 cases in stage IB, 36 cases in stage IIA, 38 cases in stage IIB, and 12 cases in stage IIIA (Table 1).

### 3.4. Univariate Analysis of Diagnosis of Benign and Malignant Nodules

Benign and malignant nodules had significant differences in patient age, maximum diameter of nodules, calcification, lobular sign, burr sign, vascular cluster sign, and pleural depression sign (*P* < 0.05). There were no significant differences in patient gender, clinical symptoms, smoking history, past tumor history, lesion location, and vacuole sign (*P* > 0.05) (Table 2).

### 3.5. Multivariate Analysis of Diagnosis of Benign and Malignant Nodules

The benign and malignant diagnostic findings were used as the dependent variable *Y* (yes = 1, no = 0), and age, maximum nodule diameter, calcification, lobarization sign, burr sign, vascular collection sign, and pleural depression sign were used as the independent variable *X* and subjected to multivariate logistic regression analysis. The assigned values are shown in Table 3. Age, maximum diameter of nodules, lobular sign, burr sign, vascular cluster sign, and pleural depression sign are independent factors related to the diagnosis of benign and malignant nodules (*P* < 0.05, Table 4).

## 4. Discussion

The pathogenesis of SPN is complex, but its occurrence often suggests the presence of early lung cancer and other diseases [8]. It is difficult to determine the benign and malignant SPN due to the large difference in clinical symptoms and imaging findings of SPN patients, and we can observe that some SPN imaging examinations show malignant signs, but the pathological diagnosis after surgery shows benign lesions [9]. Therefore, it is of great significance to improve the diagnosis efficiency of SPN benign and malignant and adopt corresponding effective treatment methods to improve the efficacy and long-term survival rate of patients [10].

VATS is a mature minimally invasive surgical technique. A number of studies [11, 12] showed that VATS is easier to be accepted by physicians and patients in the process of clinical application because it has both small wounds, light postoperative pain, and complications. The advantages are fewer symptoms and faster recovery after surgery. In this study, we retrospectively analyzed the clinical data of 317 SPN patients who underwent VATS resection and found that 124 patients (39.12%) underwent single-hole VATS and 193 patients (60.88%) underwent multi-hole VATS. Single-port operation is a further development of classic VATS under the concept of minimally invasive and rapid recovery, which has the advantages such as minimizing the incision, optimizing the field of view, and reducing chest wall and intercostal nerve injuries compared with multi-port VATS. However, single-port VATS requires more skill and experience from the surgeon [13]. Lobectomy was performed in 195 cases (61.51%), anatomical segmental lung resection in 16 cases (5.05%), and pulmonary wedge resection in 106 cases (33.44%) in this study. We performed wedge resection for benign SPN and lobectomy or segmental lung resection and lymph node dissection for malignant SPN, except for three patients who were converted to open surgery intraoperatively due to pleural atresia. This shows that both benign and malignant SPN can be diagnosed and effectively treated with VATS [14].

No serious adverse outcome events such as death occurred in any patients during the perioperative period. The three patients who underwent open-chest surgery had a mean operative time of 68.00 minutes, intraoperative blood loss of 123.33 ml, drainage tube retention time of 6.33 days, and postoperative hospital stay of 12.25 days, compared with the two groups of patients who underwent single-port VATS and multi-port VATS, all of which were at similar and lower levels. VATS treatment for benign and malignant SPN is less invasive and has fewer complications, which is conducive to the recovery of the patient's body function after surgery, and can complete the diagnosis and treatment at once, avoiding secondary surgery and long-term follow-up repeated examinations [15]. After the operation, our physicians discussed and studied many times and summarized the intraoperative experience and precautions that the choice of single-hole or multi-hole VATS should be made according to the individualized situation of the patient and the experience and level of the surgical operator. In cases where patients present with severe thoracic adhesions and difficult exposure, blind adherence to single-port VATS will not only make the procedure more difficult but also lead to prolonged anesthesia and operative time and increased postoperative complications.

All 317 patients in this study were pathologically diagnosed, of which 98 cases (30.91%) were benign nodules, including hamartoma, inflammatory pseudotumor, and tuberculoma most of which were inflammatory pseudotumor and tuberculoma. 219 cases (69.09%) were malignant nodules, including squamous cell carcinoma, adenocarcinoma, carcinoid, small cell carcinoma, large cell carcinoma, and adenosquamous carcinoma of which adenocarcinoma and squamous cell carcinoma were the main ones, accounting for 44.75% and 48.86% of malignant SPN, respectively, and TNM staging is mostly stage I. The above fully confirms that early effective treatments for SPN can achieve better treatment results while confirming the diagnosis, avoiding repeated inspections and treatment delays [16, 17].

The clinical symptoms and imaging features of benign and malignant SPN partially overlap, which brings great difficulties to clinicians in the diagnosis and treatment, and there is uncertainty. However, CT imaging features are still an important basis for diagnosis of benign and malignant nodules [18]. The results of this study show that benign and malignant nodules are significantly different in terms of patient age, nodule diameter, calcification, lobular sign, burr sign, vascular cluster sign, and pleural depression sign. And further analysis showed that age, nodule diameter, lobular sign, burr sign, vascular cluster sign, and pleural depression sign are independent factors affecting the diagnosis of benign and malignant SPN, which suggests that older patients with SPN should be more cautious to the development of early lung cancer and be promptly treated with effective surgical management or closely followed up [19]. The study by Chen et al. [20] showed that the probability of SPN being diagnosed as malignant is significantly increased when its diameter exceeds 10 mm, which suggests that the benign and malignant SPN are significantly related to the diameter of the nodule. Malignant SPN imaging usually shows a gravelly or diffuse distribution with a small extent, while benign SPN imaging shows smooth, intact margins with clear contours [21, 22]. Studies [23] have pointed out that the signs of malignant lesions in pulmonary nodules include pleural traction, burr sign, lobular sign, tumor vascular sign, bronchus truncation sign, etc., and the results of this study are generally consistent with them.

In summary, VATS is a minimally invasive procedure with few complications and is of great clinical value in the diagnosis and treatment of benign and malignant SPN. Age, nodal diameter, lobar sign, burr sign, vascular collection sign, and pleural depression sign are independent factors affecting the diagnosis of benign and malignant SPN; therefore, patients who are older and have risk factors on imaging should be given high priority and managed early and aggressively or followed up closely.

## Figures and Tables

**Figure 1:** Surgical status of patients. (a) Surgical resection status: proportion of lobectomies, anatomical segmental lung resections, and wedge lung resections. (b) Surgical method: Percentage of single-hole VATS vs. multi-hole VATS.

**Figure 2:** Comparison of the postoperative situation of patients undergoing single-port VATS operation and multi-port VATS operation. (a) Comparison of mean operative time. (b) Comparison of mean intraoperative bleeding. (c) Comparison of the mean drainage tube retention time. (d) Comparison of the mean hospital stay. (e) Comparison of postoperative complications.

**Table 1:** Postoperative pathological diagnosis of patients (*n*, %).

Pathological type and staging	Case no. (%)
Benign	98 (30.91%)
Hamartoma	12 (12.24%)
Inflammatory pseudotumor	37 (37.76%)
Tuberculoma	32 (32.65%)
Bronchogenic cyst	2 (2.04%)
Sclerosing hemangioma	9 (9.18%)
Solitary fibroma	6 (6.13%)
Malignant	219 (69.09%)
Squamous cell carcinoma	107 (48.86%)
Adenocarcinoma	98 (44.75%)
Carcinoid	1 (0.46%)
Small cell carcinoma	2 (0.91%)
Large cell carcinoma	8 (3.65%)
Adenosquamous carcinoma	2 (0.91%)
Sarcomatoid carcinoma	1 (0.46%)
TNM staging	219 (69.09%)
IA	61 (27.85%)
IB	72 (32.88%)
IIA	36 (16.44%)
IIB	38 (17.35%)
IIIA	12 (5.48%)

**Table 2:** Univariate analysis of diagnosis of benign and malignant nodules (*n*, %).

Clinical information	Benign (*n* = 98)	Malignant (*n* = 219)	*χ*^*2*^ value	*P* value
Gender	—	—	0.347	0.556
Male	52 (53.06%)	124 (56.62%)	—	—
Female	46 (46.94%)	95 (43.38%)	—	—

Age	—	—	5.688	0.001
≥45 years old	42 (42.86%)	137 (62.56%)	—	—
<45 years old	56 (57.14%)	82 (37.44%)	—	—

Clinical symptoms	—	—	1.507	0.261
Yes	55 (56.12%)	98 (44.75%)	—	—
No	43 (43.88%)	121 (55.25%)		

Smoking history	—	—	0.235	0.627
Yes	37 (37.76%)	89 (40.64%)	—	—
No	61 (62.24%)	130 (59.36%)	—	—

Past history of tumor	—	—	0.815	0.367
Yes	6 (6.12%)	20 (9.13%)	—	—
No	92 (93.88%)	199 (90.87%)	—	—

Maximum nodule diameter (mm)	—	—	4.878	0.009
≤20 mm	52 (53.06%)	84 (38.36%)	—	—
21–30 mm	46 (46.94%)	135 (61.64%)	—	—

Lesion site	—	—	0.527	0.459
Upper lobe of right lung	35 (35.71%)	61 (27.85%)	—	—
Middle lobe of right lung	12 (12.24%)	19 (8.68%)	—	—
Lower lobe of the right lung	17 (17.35%)	41 (18.72%)	—	—
Upper lobe of the left lung	19 (19.39%)	60 (27.40%)	—	—
Lower lobe of left lung	15 (15.31%)	38 (17.35%)	—	—

Calcification	—	—	4.168	0.016
Yes	23 (23.47%)	3 (1.37%)	—	—
No	75 (76.53%)	216 (98.63%)	—	—

Lobarization sign	—	—	3.824	0.019
Yes	11 (11.22%)	168 (76.71%)	—	—
No	87 (88.78%)	51 (23.29%)	—	—

Burr sign	—	—	4.018	0.017
Yes	36 (36.73%)	172 (78.54%)	—	—
No	53 (54.08%)	47 (21.46%)	—	—

Vascular cluster sign	—	—	4.681	0.010
Yes	4 (4.08%)	72 (32.88%)	—	—
No	94 (95.92%)	147 (67.12%)	—	—

Vacuolation sign	—	—	2.042	0.183
Yes	12 (12.24%)	39 (17.81%)	—	—
No	86 (87.76%)	180 (82.19%)	—	—

Pleural depression sign	—	—	3.594	0.021
Yes	18 (18.37%)	174 (79.45%)	—	—
No	80 (81.63%)	45 (20.55%)	—	—

**Table 3:** Assigned values for multivariate analysis factors.

Factors	Assignment
Age	≥45 = 0, <45 = 1
Maximum nodule diameter	≤20 = 0, 21–30 = 1
Calcification	Yes = 0, no = 1
Lobarization sign	Yes = 0, no = 1
Burr sign	Yes = 0, no = 1
Vascular clustering sign	Yes = 0, no = 1
Pleural depression sign	Yes = 0, no = 1

**Table 4:** Multivariate analysis of diagnosis of benign and malignant nodules.

Factors	*B*	SE	Wald's	df	Sig.	Exp (B)
Age	1.956	0.341	3.594	1	0.042	2.168
Maximum nodule diameter	2.384	0.284	5.168	1	0.038	1.528
Calcification	1.527	0.276	2.517	1	0.153	1.276
Lobarization sign	3.025	0.246	4.861	1	0.026	1.864
Burr sign	2.964	0.218	5.108	1	0.029	1.093
Vascular clustering sign	2.168	0.294	6.358	1	0.012	1.166
Pleural depression sign	2.457	0.179	6.127	1	0.023	1.584

## Data Availability

The data used during the current study are available from the corresponding author and the Department of Academic Research, the First Medical Center of Chinese PLA General Hospital on reasonable request.
